This article has been retracted.

# Development and Validation of a Postoperative Delirium Prediction Model for Elderly Orthopedic Patients in the Intensive Care Unit

**DOI:** 10.1155/2021/9959077

**Published:** 2021-06-08

**Authors:** Gang Wang, Lei Zhang, Ying Qi, Guangjian Chen, Juan Zhou, Huihui Zhu, Yingxin Hao

**Affiliations:** ^1^Department of Critical Care Medicine, Tongji Hospital, Tongji University School of Medicine, Tongji University, Shanghai 200065, China; ^2^Department of Economic Management, Yingkou Institute of Technology, Yingkou 115014, Liaoning, China

## Abstract

We developed a prediction model for delirium in elderly patients in the intensive care unit who underwent orthopedic surgery and then temporally validated its predictive power in the same hospital. In the development stage, we designed a prospective cohort study, and 319 consecutive patients aged over 65 years from January 2018 to December 2019 were screened. Demographic characteristics and clinical variables were evaluated, and a final prediction model was developed using the multivariate logistic regression analysis. In the validation stage, 108 patients were included for temporal validation between January 2020 and June 2020. The effectiveness of the model was evaluated through discrimination and calibration. As a result, the prediction model contains seven risk factors (age, anesthesia method, score of mini-mental state examination, hypoxia, major hemorrhage, level of interleukin-6, and company of family members), which had an area under the receiver operating characteristics curve of 0.82 (95% confidence interval 0.76–0.88) and was stable after bootstrapping. The temporal validation resulted in an area under the curve of 0.80 (95% confidence interval 0.67–0.93). Our prediction model had excellent discrimination power in predicting postoperative delirium in elderly patients and could assist intensive care physicians with early prevention.

## 1. Introduction

Delirium, which is defined as an acute disorder of attention and cognition, is a common, life-threatening, and preventable clinical syndrome in older persons. The etiopathogenesis of delirium remains unclear [1]. Delirium often occurs after severe disease, surgery, or hospitalization and is often overlooked by clinicians. The development of delirium initiates a serious range of events culminating in loss of independence, increased morbidity and mortality, institutionalization, and catastrophic medical costs [2, 3]. Each year, more than 2.6 million adults over 65 years develop delirium, accounting for an estimated expenditure over $164 billion in annual healthcare in the United States [4].

Delirium is one of the most common surgical complications among older patients, the incidence of which is between 15 and 25% after major elective procedures and approximately 50% after high-risk surgeries such as hip fracture repair and cardiac surgery [5]. The cumulative incidence of delirium exceeds 75% in patients undergoing mechanical ventilation in the intensive care unit (ICU) [6]. Because of its adverse effects on function and quality of life, delirium has significant societal implications for individuals, families, communities, and entire healthcare system.

To date, there is no convincing evidence that pharmacological prevention or treatment is effective, and multicomponent nonpharmacological risk factor-controlled approaches have proven to be the most effective strategies for reducing the incidence of delirium [7]. General preventive measures for all intensive care patients is time-consuming, and a number of patients may be exposed to unnecessary risks, such as the adverse effects of drug prophylaxis. There are two predictive models for intensive care patients [8, 9], with an area under the receiver operating characteristic (AUROC) curve of 0.77 (95% CI, 0.74–0.79) and 0.76 (95% CI, 0.73–0.77), respectively. Both prediction models, with focus on medical inpatients, had similar predictive values based on screening with the confusion assessment method for the ICU (CAM-ICU) [10]. In clinical practice, however, the predictive value is not satisfactory for surgical patients, especially for critical care patients after orthopedic surgery. The aim of our study was to develop a new delirium prediction model for older patients in the ICU after orthopedic surgery and validate as well as evaluating its effectiveness.

## 2. Materials and Methods

### 2.1. Study Design

This was an observational study in which we developed a prediction model for delirium in elderly patients in the ICU who underwent orthopedic surgery and then temporally validated it in a second prospective cohort in the same hospital. The inclusion criteria and study protocol were the same for both recruited groups. The study protocol was approved by the Clinical Research Ethics Committee of Tongji Hospital (2018-TJDX-176). The study protocol, including potential risks and benefits, was explained to patients in person before we obtained written informed consent from the patients or their legal representatives.

### 2.2. Study Population for Development and Validation Studies

We conducted a prospective cohort study at Tongji Hospital to develop a prediction model. Between January 2018 and December 2019, a total of 506 elderly patients in the ICU who underwent orthopedic surgery were screened, 319 of whom were finally included in the analyses. We included all adult patients, aged 65 years or older, who were admitted to the ICU after orthopedic surgery. We excluded patients who were delirious before admission to the ICU, stayed in the ICU for less than 24 h, were mechanically ventilated, had serious auditory or visual disorders, were severely mentally disabled, were unable to provide informed consent, or had the compliance rate of the delirium screening less than 80% during the ICU stay.

We conducted a second prospective cohort study for temporal validation of the model between January 2020 and June 2020 in the same hospital, and 108 patients were included.

### 2.3. Risk Factors

We collected demographic variables, mini-mental state examination (MMSE), and Charlson Comorbidity Index score before admission to the ICU. Information on mode of anesthesia, operative duration, bleeding volume, hypotension and hypoxia during the operation, company of family members during a patient's stay in the ICU, and serum concentration of interleukin-6 (IL-6) were also recorded within 2 h after admission to the ICU. Hypoxia was defined as SpO_2_ (oxygen saturation) less than 90% at any time during the entire operation. Hypotension was defined as a patient's mean arterial pressure less than 65 mmHg at any time or vasopressor agents were administered, regardless of the duration. Company of family members implied that at least one family member accompanied the patient for more than 6 h during the night. A total loss of more than 400 ml of blood was considered a major hemorrhage. We excluded patients under mechanical ventilation from our study. Hence, sedative agents (e.g., midazolam or dexmedetomidine) were not routinely administered unless RASS score was more than 2 points. Continuous patient-controlled intravenous analgesia or regional analgesia was provided to relieve postoperative pain. When necessary, all enrolled patients were sedated and anesthetized using the same protocol.

To detect delirium, all consecutive intensive care patients were screened at least three times daily. When required, for example, after sudden changes in behavior, attention, or consciousness, an additional assessment was performed. All research nurses and physicians received training for delirium assessment, and the use of the CAM-ICU tool before the study was initiated.

### 2.4. Outcome Definition

The main outcome was the development of delirium within 24 h during the patients' stay in the ICU. Patients with delirium were defined as those who had at least one positive CAM-ICU screening during their stay in the ICU. In addition, if the clinical presentation provided signs of delirium without a positive CAM-ICU screening, or conversely, if the clinical presentation did not provide evidence of delirium and the patient had a positive CAM-ICU result, a senior psychiatrist was informed to confirm the diagnosis of delirium and rule out false negatives and false positives using the Diagnostic and Statistical Manual of Mental Disorders, fourth edition diagnostic criteria [11]. All patients with diagnosis confirmed by a psychiatrist were assigned to the delirium group.

### 2.5. Statistical Analysis

In previous studies, the incidence of delirium in intensive care patients was approximately 28%. We calculated the sample size based on the need for 10 delirious patients per risk factor plus 5% dropout for the prediction development of the model. Consequently, at least 300 patients were required to develop the model. The data from the temporal validation study for all variables were complete. Risk factors were collected as continuous, categorical, or dichotomized variables.

In our study, continuous variables were expressed as medians with standard deviations (SDs), and categorical data were expressed as percentages. The independent Student's t-test or Mann–Whitney U test was used to compare continuous variables when appropriate, and the chi-square test or Fisher's exact test was used to compare categorical variables with or without delirium. We used univariate logistic regression to assess the association between each potential prognostic determinant and the presence or absence of delirium. We excluded determinants with a prevalence rate below 10%, or with a *p* value above 0.10, in univariate analysis. With the remaining significant variables detected by univariate analysis (*p* value <0.10), we used the multivariate regression analysis to evaluate the independent associations with the occurrence of delirium. The predictive accuracy of this model was evaluated using the AUROC curve. Bootstrapping techniques were used to balance for overfitting, and 500 random bootstrap samples resulted in shrunken regression coefficients of the risk factors and the AUROC curve of the final developed model.

In the validation study, we multiplied each shrunken regression coefficient by the value of each risk factor, and the calculated result was the predicted probability with which we built a new AUROC curve. The Youden index (the maximum sum of sensitivity and specificity is 1) was used to determine the optimal cutoff point of the prediction model. Finally, a calibration plot was used to evaluate the agreement between the predicted probability and actual outcome. A calibration slope of 1 and an intercept of 0 indicated ideal calibration. A calibration belt plot consisting of a calibration curve with 95% confidence interval (CI) was designed to illustrate the relationship between predicted probabilities and actual probabilities by fitting a polynomial logistic analysis. When the bisector vector did not cross the calibration belt, a significant statistical deviation from the bisector occurred, and the *p* value (*p* < 0.05) indicated that the calibration of the prediction model was not perfect. All statistical analyses were performed using *R* statistics version 3.0.1 and SPSS 16.01. Statistical significance was set at a two-sided *p* value of <0.05.

## 3. Results

### 3.1. Development of Prediction Model

In the development cohort, 319 consecutive patients were included, 85 of which (26.6%) developed delirium within 24 h.  Table 1 shows the patients' demographic characteristics, surgery-related risk factors, and other potential risk factors. By comparing the characteristics and potential risk factors between patients who developed postoperative delirium (POD) and those who did not, in the univariate logistic regression analysis, we found that patients who underwent surgery with delirium had significant differences in age, anesthesia method, MMSE score, hypoxia during surgery, company of family members during ICU, serum concentration of IL-6 above 9 ng/ml, and major hemorrhage (*p* < 0.10). Hypertension, Charlson comorbidity index, urgent admission, and duration of surgery were removed because of a *p* value >0.10.

Table 2 summarizes the values or percentages of patients with each risk factor and the odds' ratio with a 95% confidence interval for delirium. The remaining seven risk factors entered into the multivariate logistic regression analysis, and we constructed a final prediction model. The AUROC curve of the prediction model was 0.82 (95% CI, 0.76 to 0.88) and did not change noticeably after bootstrapping (Figure 1). Based on the ROC analysis of the development population, we calculated the result of Youden index as 0.56, and at this optimal cutoff point, the sensitivity and specificity were 0.74 and 0.82, respectively.

### 3.2. Temporal Validation of Prediction Model

In the prospective validation study, we screened 108 consecutive patients and all data were complete. 18 of the validation patients (16.7%) developed delirium. The temporal validation resulted in an AUROC curve of 0.80 (95% CI 0.67 to 0.93).  Figure 2 shows the calibration curves of the validation cohort.

## 4. Discussion

Delirium is common in elderly orthopedic patients in the ICU and is associated with worse outcomes. Although there is insufficient evidence to show that pharmacologic prevention or treatment is effective, clinicians prefer atypical antipsychotic agents to prevent or treat postoperative delirium [12]. Much more research has suggested that a multicomponent, nonpharmacological intervention significantly reduces delirium [13, 14]. However, medical resources were extremely limited, and it was difficult to guarantee that each patient was treated with adequate preventive measures, especially in the ICU.

A previous prediction model with ten risk factors (age, admission group, urgent admission, sedation, morphine use, infection, coma, APACHE-II score, urea level, and metabolic acidosis) had an AUROC curve of 0.77 (95% CI, 0.74–0.79). This model did not reflect the impact of surgery-related risk factors on POD, which had a good predictive value in medical patients instead of surgical patients. In addition to demographic characteristics, surgery, anesthesia-related risk factors, and inflammatory factors were also included in our study. Finally, we developed a predictive model of seven risk factors (age, anesthetized method, MMSE score, hypoxia during operation, company of family members, serum concentration of IL-6 above 9 ng/ml, and major hemorrhage). For elderly people in the ICU who underwent an orthopedic procedure, the model had an excellent prediction power with an AUROC of 0.82 (95% CI, 0.76 to 0.88).

Capri et al. [15] found that the preoperative level of IL-6 was significantly associated with POD in elderly patients. High IL-6 plasma level (specifically >9 pg/mL) was an independent risk factor for delirium onset (odds' ratio (OR): 4.9; 95% CI, 1.6–14.63; *p* < 0.001). Growing evidence indicates that circulating levels of cytokines may influence the function of the cerebral nervous system [16]. Another study found higher IL-6 immunoreactivity in the brain of patients with delirium, which suggested a close association between human brain activity of microglia, IL-6, and delirium in elderly patients [17]. To date, there is no model with IL-6 to predict the incidence of delirium because the level of IL-6 has not been routinely tested in orthopedic wards or ICUs. During the first few days after the operation, patients' cognitive function decreased significantly in patients who received general anesthesia (*p* < 0.001) compared to those who received regional anesthesia [18]. Interestingly, in a previous study the impact of the anesthesia method on the incidence of postoperative delirium was not significant between regional and general anesthesia [19]. Possible reasons include the small sample size, substantial heterogeneity regarding study design, delirium assessment tools, assessment time points, and anesthetic protocol. There is an urgent need to ascertain the impact of anesthesia methods on the outcomes of delirium with methodologically rigorous research. In our study, we found that general anesthesia was an independent risk factor for POD.

ICU physicians in Tongji Hospital calculated the probability of POD through the multivariate regression equation and combined this with their clinical experience to determine the optimal individualized cutoff value for initiating prophylactic measures. For patients at high risk of delirium, more active and adequate prevention measures would be provided, which not only optimizes the limited medical resources but also improves the patients' health. The prognosis may also enable patients to avoid adverse events due to drug exposure.

There are several limitations to our study. First, the sample size of the development model cohort was relatively small. Seven risk factors were included in the final prediction model, and the incidence of delirium in the development population in this study was 26.6%. Based on the need for ten positive results per risk factor, at least 290 patients were needed. The sample size met the minimum requirements. Second, we did not conduct a prospective cohort study for external validation despite the use of bootstrapping procedures to balance the capabilities of the prediction model, which may overestimate the diagnostic power when performed in other hospitals. Third, a low dose dexmedetomidine infusion significantly decreased the incidence of delirium in the first few days after surgery in elderly patients admitted to the ICU [20, 21]. In our study, some patients with regional block anesthesia were administered dexmedetomidine, resulting in a reduced incidence of postoperative delirium. This may expand the effect of anesthesia on predicting postoperative delirium. Finally, the delirium prediction model may not be appropriate for patients with serious auditory or visual disorders because they were not included in our study.

## 5. Conclusions

Our prediction model had excellent discrimination in predicting postoperative delirium in elderly patients and could assist intensive care physicians in initiating early prevention.

## Figures and Tables

**Figure 1:** AUROC curve of the development cohort.

**Figure 2:** Calibration plot of the validation cohort.

**Table 1:** The demographic characteristics and clinical variables of the development and validation cohorts.

	Development cohort	Validation cohort
Patients (*n*)	319	108
Male sex (*n*) (%)	206 (64.6)	65 (60.2)
Age (years) (mean ± SD)	83.1 ± 7.9	80.1 ± 8.4
BMI (kg/m^2^) (mean ± SD)	23.3 ± 3.0	23.5 ± 2.8
Urgent admission (*n*) (%)	110 (34.5)	31 (28.7)
MMSE (mean ± SD)	20.1 ± 4.2	20.5 ± 4.1
Charlson comorbidity index (mean ± SD)	7.4 ± 3.1	8.4 ± 3.4
Duration of surgery (min) (mean ± SD)	148.0 ± 52.4	110.4 ± 36.7
Regional anesthesia (*n*) (%)	166 (52)	58 (53.7)
Hypotension during surgery (*n*) (%)	85 (26.6)	17 (15.7)
Hypoxia during surgery (*n*) (%)	42 (13.2)	15 (13.9)
Major hemorrhage (*n*) (%)	109 (34.2)	37 (34.3)
Level of IL-6 >9pg/ml (*n*) (%)	112 (35.1)	45 (41.7)
Company of family member (*n*) (%)	109 (34.2)	43 (39.8)

BMI denotes body mass index, MMSE denotes mini-mental state examination, SD denotes standard deviation, and IL-6 denotes interleukin-6.

**Table 2:** Univariate logistic regression analyses and the final multivariate logistic regression model in the development cohort.

Variables	Univariate			Coefficient	Multivariate		
	OR	*p*	95% CI		OR	*p*	95% CI
Age	1.093	<0.001	1.055–1.133	0.085	1.089	<0.001	1.046–1.133
MMSE	0.839	<0.001	0.784–0.897	−0.186	0.83	<0.001	0.768–0.897
Regional anesthesia	0.482	0.005	0.290–0.800	−0.733	0.481	0.016	0.264–0.874
Hypoxia during surgery	2.09	0.032	1.065–4.101	0.845	2.327	0.045	1.020–5.310
Major hemorrhage	1.62	0.064	0.972–2.702	0.531	1.701	0.092	0.917–3.157
Level of IL-6 >9pg/ml	3.446	<0.001	2.056–5.774	1.313	3.719	<0.001	2.036–6.793
Company of families	0.59	0.062	0.339–1.026	−0.743	0.476	0.026	0.247–0.916

MMSE denotes mini-mental state examination, OR denotes odds' ratio, and CI denotes confidence interval.

## Data Availability

The data used to support the study are available from the corresponding author upon request.
